The article "High‐intensity focused ultrasound inhibits invasion and metastasis of colon cancer cells by enhancing microRNA‐124‐mediated suppression of STAT3" was retracted in 2022. Reasons: duplicated images; signs of a paper mill.

# High‐intensity focused ultrasound inhibits invasion and metastasis of colon cancer cells by enhancing microRNA‐124‐mediated suppression of STAT3

**DOI:** 10.1002/2211-5463.12642

**Published:** 2019-05-04

**Authors:** Meiying Li, Guangsheng Wan, Hongjie Yu, Wei Xiong

**Affiliations:** ^1^ Department of Ultrasound Shanghai University of Traditional Chinese Medicine Affiliated PUTUO Hospital China; ^2^ Oncology Department of Traditional Chinese Medicine Shanghai University of Traditional Chinese Medicine Affiliated PUTUO Hospital China

**Keywords:** colorectal cancer, high‐intensity focused ultrasound, metastasis, miR‐124, STAT3

## Abstract

Metastasis is the primary contributor to colorectal cancer mortality. High‐intensity focused ultrasound (HIFU) is an emerging technology for tumor therapy that exerts its effects through tumor ablation, mechanical disruption, and enhancement of immune responses. However, it remains unclear whether HIFU can influence tumor metastasis. Here, we examined the effect of HIFU on tumor metastasis of colorectal cancer cells and the underlying mechanisms. HIFU was observed to inhibit migration of HCT‐116 cells *in vitro* and suppress lung metastasis in a mouse model of colon cancer. In addition, HIFU up‐regulated microRNA (miR) ‐124 expression, which inhibited the activation of signal transducer and activator of transcription 3 (STAT3) and inhibited migration of HCT‐116 cells. Treatment with an inhibitor of miR‐124 reversed the effect of HIFU on cell migration. In conclusion, our results suggest that HIFU exerts anti‐metastatic effects in colon cancer, and this effect is possibly mediated via up‐regulation of miR‐124 and subsequent miR‐124‐mediated STAT3 suppression.

**Abbreviations**
GAPDH: glyceraldehyde 3‐phosphate dehydrogenase
HIFU: high‐intensity focused ultrasound
JAK: Janus kinase
miRNA: microRNA
MTT: 3‐(4,5‐dimethylthiazol‐2‐yl)‐2,5‐diphenyl‐tetrazolium bromide
PI: propidium iodide
STAT3: signal transducer and activator of transcription 3
3′‐UTR: 3′‐untranslated region

Colorectal cancer is a malignant cancer that can spread to or invade other parts of the body at advanced stages. Metastasis of colorectal cancer is a main contributor to the mortality of this disease. In patients at an early stage of colorectal cancer, the 5‐year survival rate is more than 90%, compared with 10–15% in patients with distant metastases 1. Therefore, research into new techniques for inhibiting invasion and metastasis of colorectal cancer is of great significance for the treatment of this disease.

High‐intensity focused ultrasound (HIFU) is an emerging technology for cancer therapy. It can have both a thermal and a non‐thermal effect and result in ablation or mechanical disruption of target tissues 2. After more than 10 years of development, this therapy has been widely studied in clinical trials in treating benign or malignant tumors in various organs, including liver, pancreas, breast, kidney and thyroid 2. Besides the effect of tissue ablation and mechanical disruption, HIFU is also found to enhance the anti‐cancer immune responses 3. A recent study found that HIFU could inhibit melanoma metastasis through inhibiting the microRNA (miRNA)‐21 pathway 4. However, whether HIFU has an effect on the invasion and metastasis of colorectal cancer remains unclear.

The article "High‐intensity focused ultrasound inhibits invasion and metastasis of colon cancer cells by enhancing microRNA‐124‐mediated suppression of STAT3" was retracted in 2022. Reasons: duplicated images; signs of a paper mill.

MiRNAs are a class of non‐coding regulatory RNAs of 18–25 nucleotides in length that play a role in cancer; more specifically, a family of miRNAs termed metastamirs have been shown to control metastatic progression 5, 6. In colorectal cancer, the expression of several miRNAs is altered, and the altered expression patterns are associated with various pathogenetic signaling pathways 7. MiR‐124 is one of those miRNAs that are involved in colorectal cancer. Previous studies found decreased miR‐124 mRNA expression in clinical samples of colorectal cancer patients 8. *In vitro* studies found that miR‐124 could inhibit cell metastasis and invasion of colorectal cancer 9. A recent study found that focused ultrasound treatment in rats increased the plasma abundance of several miRNAs 10. Here we speculated that HIFU could regulate invasion and metastasis of colorectal cancer by causing alterations of miRNA expression.

## Materials and methods

### Cell culture and HIFU treatment

HCT‐116 human colon cancer cells (ATCC, Manassas, VA, USA) were cultured in RPMI‐1640 medium with 10% FBS (Invitrogen, Carlsbad, CA, USA), l‐glutamine (2 mm), streptomycin (100 μg·mL^−1^) and penicillin (100 U·mL^−1^) (Beyotime Biotechnology, Shanghai, China) in 5% CO_2_ at 37 °C.

For HIFU treatment, cells at logarithmic phase of growth were resuspended in medium in 1.5 mL polyethylene centrifuge tubes at a density of 2 × l0^6^ cells/tube. The ultrasound waves were generated by a HIFU apparatus (Haifu Medical Technology, Chongqing, China) and the energy was focused at the center of the tube. Cells received HIFU treatment at an intensity of 142.7 W·cm^−2^ for 1, 2 or 3 s.

### Measurement of cell migration

For a wound healing assay, cells were seeded and cultured in six‐well plates after HIFU treatment. For each well a scratch wound was made by a pipette tip in the middle of the bottom. Then the wells were washed with medium to remove the detached cells, and culture continued for an additional 48 h. The gap closure rate = (1–48 h gap width/0 h gap width) × 100%.

The article "High‐intensity focused ultrasound inhibits invasion and metastasis of colon cancer cells by enhancing microRNA‐124‐mediated suppression of STAT3" was retracted in 2022. Reasons: duplicated images; signs of a paper mill.

Transwell chambers (8 μm pore size; Corning Costar, Corning, NY, USA) were used to perform a Transwell migration assay. RPMI‐1640 medium with 20% FBS was added to the lower chamber as a chemo‐attractant and cells were plated in the upper membrane. After 48 h, cells on the lower chamber were fixed with 4% paraformaldehyde, stained with crystal violet, and the number of cells was manually counted under a microscope at ×100 magnification from five randomly selected visual fields.

### Trypan Blue exclusion assay

After HIFU treatment, cells were cultured for an additional 48 h. Then cells were resuspended, stained with Trypan Blue (Beyotime Biotechnology) and counted using a hemocytometer under a light microscope.

### MTT assay

After HIFU treatment, cells were cultured in 96‐well plates for an additional 48 h. Then a 3‐(4,5‐dimethylthiazol‐2‐yl)‐2,5‐diphenyl‐tetrazolium bromide (MTT) assay was carried out using the MTT reagent (Promega, Madison, WI, USA), following the manual. The absorbance was measured at 492 nm.

### Apoptosis assay

After HIFU treatment, cells were cultured in six‐well plates for an additional 48 h. Then apoptosis was assessed using a commercial annexin V/propidium iodide (PI) staining kit (Beyotime Biotechnology) following the manual. Annexin V^+^/PI^−^ cells were defined as apoptotic cells by flow cytometry (Beckman Coulter, Indianapolis, IN, USA).

### Transfection and luciferase assay

HCT‐116 cells were transfected with miR‐124, the negative control (miR‐124 NC) or miR‐124 inhibitor (AMO‐miR‐124) (all purchased from Life Technologies, Carlsbad, CA, USA) using Lipofectamine RNAiMAX (Life Technologies). Cells were harvested 48 h later and mRNA expression and the protein level of signal transducer and activator of transcription 3 (STAT3) were measured.

For luciferase assay, the whole 3′‐untranslated region (3′‐UTR) of STAT3 and the mutated 3′‐UTR of STAT3 were cloned into psiCHECK2 vectors. After HIFU treatment, cells were co‐transfected with the reporter vectors and miR‐124 mimics or inhibitors. pRL‐TK *Renilla* luciferase vectors were also co‐transfected as an internal control. After 48 h, cells were lysed and luciferase activity was measured with the Dual Luciferase Reporter System (Promega).

### Animal model of colon cancer and HIFU treatment

To establish the colon cancer transplant model, HCT‐116 cells were subcutaneously injected into the axilla of nude mice (2 × l0^7^ cells/mouse). Tumor size was measured using digital calipers every day. When the tumors reached 7–8 mm in diameter, mice were divided into two groups and subjected to HIFU treatment or sham treatment. The ultrasound waves were generated by a Seapostar HIFU apparatus (Haifu Medical Technology) with parameter of 9.3 MHz and 4.5 W. Treatment started at the center of the tumor and gradually expanded to the border with a step size of 1.0 mm and 10 s exposure for each treated spot. Mice were sacrificed 7 weeks later. To count the metastatic lung nodules, lung tissues were stained with Bouin's solution. The remaining lung tissues were used for qRT‐PCR and western blot analyses. The animal study was approved by Shanghai University of Traditional Chinese Medicine Affiliated PUTUO Hospital.

The article "High‐intensity focused ultrasound inhibits invasion and metastasis of colon cancer cells by enhancing microRNA‐124‐mediated suppression of STAT3" was retracted in 2022. Reasons: duplicated images; signs of a paper mill.

### qRT‐PCR

Total RNA was extracted from HIFU‐treated HCT‐116 cells or mouse lung tissues. Quantitative RT‐PCR was carried out using the One‐Step TB Green PrimeScript Kit (Takara, Dalian, China). The relative mRNA level was calculated using the $2^{-\Delta \Delta C_{t}}$ method. The primers were: human *STAT3*: 5′‐GCCAGAGAGCCAGGAGCA‐3′ and 5′‐ACACAGATAAACTTGGTCTTCAGGTATG‐3′; human glyceraldehyde 3‐phosphate dehydrogenase (*GAPDH*): 5′‐CGCTCTCTGCTCCTCCTGTT‐3′ and 5′‐CCATGGTGTCTGAGCGATGT‐3′; mouse *STAT3*: 5′‐CAATACCATTGACCTGCCGAT‐3′ and 5′‐GAGCGACTCAAACTGCCCT‐3′; mouse *GAPDH*: 5′‐ATCACCATCTTCCAGGAGCG‐3′ and 5′‐TTCTGAGTGGCAG TGAGGGC‐3′. The primers for the miR‐124 and the internal control U6 snRNA were obtained from Exiqon (Woburn, MA, USA).

### Western blotting

Total protein was extracted from HIFU‐treated HCT‐116 cells or mouse lung tissues, and subjected to SDS/PAGE. A western blot assay was carried out following standard procedures. The primary antibodies were: anti‐phospho STAT3 (Tyr‐705) (1 : 800) and anti‐STAT3 (1 : 1000; Cell Signaling Technology, Danvers, MA, USA). Anti‐GAPDH (1 : 1000; Abcam, Cambridge, MA, USA) was used as internal control.

### Statistics

Data are shown as the mean ± standard error of mean (SEM). All studies were repeated in triplicate. Differences between two groups were compared by Student's *t*‐test and differences among several groups were compared by one‐way ANOVA. *P* < 0.05 was considered significant.

## Results

### HIFU exposure inhibits migration of HCT‐116 cells

As shown in Fig. 1, results of a wound healing assay showed that the percentage of gap closed was significantly lower in cells exposed to HIFU than that in control cells (Fig. 1A,B). In a transwell migration assay, the HIFU groups had significantly fewer migrated cells than the control group (Fig. 1C,D). These results showed that HIFU exposure could inhibit HCT‐116 cell migration. On the other hand, cell viability and apoptosis were not influenced by HIFU exposure (Fig. 1E–G).

**Figure 1:** HIFU exposure inhibited migration in human colon cancer HCT‐116 cells. (A, B) Wound healing assay for analyzing the effect of HIFU on migration of HCT‐116 cells. Scale bar, 100 μm. The incision width of different sites was measured, and average healing rate was calculated. *P < 0.05, **P < 0.001. Representative images are shown in (A), and average healing rate is shown in (B). (C, D) Cell migration was detected by Transwell migration assay. Scale bar, 50 μm. Representative images are shown in (C), and three independent experiments are quantified in (D). *P < 0.05, **P < 0.001. (E) Cell survival determined by Trypan Blue exclusion assay. (F) Cell viability was measured using the MTT assay. (G) The percentage of cells undergoing apoptosis measured by flow cytometry analysis. Data show mean ± SEM. One‐way ANOVA. Independent experiments were repeated in triplicate.

The article "High‐intensity focused ultrasound inhibits invasion and metastasis of colon cancer cells by enhancing microRNA‐124‐mediated suppression of STAT3" was retracted in 2022. Reasons: duplicated images; signs of a paper mill.

### HIFU exposure increases miR‐124 and decreases STAT3

qPCR showed that miR‐124 mRNA was significantly increased after HIFU exposure (Fig. 2A), while the STAT3 mRNA expression was significantly decreased (Fig. 2B), compared with those in control cells. HIFU‐treated cells showed significantly lower STAT3 and phosphorylated STAT3 (Tyr‐705) (p‐STAT3) protein levels than did control (Fig. 2C,D), indicating that HIFU could regulate miR‐124 and STAT3 in HCT‐116 cells.

**Figure 2:** HIFU exposure increased miR‐124 expression and decreased STAT3 expression in HCT‐116 cells. (A) miR‐124 expression was detected by qPCR during HIFU exposure in HCT‐116 cells. (B) STAT3 mRNA expression was detected by qPCR during HIFU exposure in HCT‐116 cells. (C, D) STAT3 protein expression was detected by western blot during HIFU exposure in HCT‐116 cells. Data show mean ± SEM. *P < 0.05, **P < 0.001 *vs* control. One‐way ANOVA. Independent experiments were repeated in triplicate.

### MiR‐124 targets and regulates STAT3

As shown in Fig. 3, STAT3 mRNA, STAT3 and p‐STAT3 protein levels in HCT‐116 cells were significantly down‐regulated in miR‐124‐transfected cells and were significantly increased in AMO‐miR‐124‐transfected cells (Fig. 3A,B). The results of a luciferase assay showed that miR‐124 suppressed the luciferase activity of STAT3 3′‐UTR but not mutated STAT3 3′‐UTR (Fig. 3C,D). These data suggested that STAT3 could be directly regulated by miR‐124 in HCT‐116 cells.

**Figure 3:** Experimental establishment of STAT3 as a target of miR‐124. (A, B) Delivery of miR‐124 significantly decreased the mRNA and protein expression levels in HCT‐116 cells. *P < 0.05, **P < 0.001 *vs* control. (C, D) miR‐124 targeting STAT3 was validated using a dual‐luciferase reporter assay. Data show mean ± SEM. **P < 0.001 *vs* miR‐124 NC. One‐way ANOVA. Independent experiments were repeated in triplicate.

### MiR‐124 inhibits migration in HCT‐116 cells

Results showed that miR‐124 significantly reduced the gap closure rates in a wound healing assay (Fig. 4A,B) and reduced the number of migrated cells in a transwell migration assay (Fig. 4C,D) in both control cells and cells exposed to HIFU, while miR‐124 inhibitor significantly increased the gap closure rates and the number of migrated cells (Fig. 4A,D) in cells exposed to HIFU. These results indicated that the effect of HIFU in inhibiting cell migration might be via miR‐124.

The article "High‐intensity focused ultrasound inhibits invasion and metastasis of colon cancer cells by enhancing microRNA‐124‐mediated suppression of STAT3" was retracted in 2022. Reasons: duplicated images; signs of a paper mill.

**Figure 4:** HIFU exposure and miR‐124 inhibited migration in human colon cancer HCT‐116 cells. (A, B) Wound healing assay for analyzing the effect of HIFU and miR‐124 on migration of HCT‐116 cells. Scale bar, 100 μm. The incision width of different sites was measured, and average healing rate was calculated. *P < 0.05 *vs* respective control group, ^#^ *P* < 0.05 *vs* respective miR‐124 group. Representative images are shown in (A), and average healing rate is shown in (B). (C, D) Cell migration was detected by Transwell migration assay. Scale bar, 500 μm. Representative images are shown in (C), and three independent experiments are quantified in (D). Data show mean ± SEM. *P < 0.05 *vs* respective control group, ^#^ *P* < 0.05 *vs* respective miR‐124 group. One‐way ANOVA. Independent experiments were repeated in triplicate.

### HIFU exposure suppresses lung metastasis of colon cancer in mice

Results of *in vivo* experiments showed that the HIFU‐treated group had significantly fewer metastatic lung nodules than the control group (Fig. 5A,B). We also found that compared with control, the HIFU‐treated group showed significantly increased miR‐124 mRNA and decreased STAT3 expression in lung tissues (Fig. 5C). STAT3 and p‐STAT3 (Tyr‐705) protein levels in the HIFU‐treated group were significantly lower than those of control (Fig. 5D). These results indicated that HIFU could suppress lung metastasis of mouse colon cancer, through increasing miR‐124 and inhibiting STAT3 signaling.

**Figure 5:** HIFU exposure suppressed lung metastasis of mouse colon cancer through attenuating miRNA‐124‐mediated STAT3 suppression *in vivo*. (A) Lungs in the treatment groups had smaller nodules. (B) The number of metastatic lung nodules decreased significantly in all treatment groups. (C) mRNA expression of miRNA‐124 and STAT3 was detected by qPCR. (D) The protein expression of STAT3 was detected by western blot. Data show mean ± SEM. **P < 0.001 *vs* control, *n* = 6 mice per group. Student's *t*‐test Independent experiments were repeated in triplicate.

## Discussion

The present study explored the effect of HIFU in tumor metastasis. HIFU is a widely studied non‐invasive technology for treatment of tumors, through tumor ablation and mechanical disruption as well as enhancing the anti‐cancer immune responses. Preliminary studies and clinical trials have been carried out to assess the possibility and effectiveness of using HIFU in treating colorectal tumors. A phase I–IIa clinical trial in patients with colorectal liver metastases showed that HIFU was a safe and effective method for tissue ablation 11. Results from animal and preclinical studies have found that HIFU induces hyperthermia in rectal targets, which could sensitize tumors to radiation and chemotherapy 12. Here we found that besides these direct thermal effects, HIFU could also inhibit migration of HCT‐116 cells and suppress lung metastasis in a mouse model of colon cancer, suggesting an effect of HIFU in reducing distant metastasis of cancers. However, results are inconsistent in different studies. A study in a mouse melanoma model found that HIFU decreased metastasis rates 13, while another study showed that pulsed‐exposure of HIFU slightly (but not significantly) increased metastasis 14. This discrepancy might be due to the different patterns of HIFU exposure, which needs further investigation.

The article "High‐intensity focused ultrasound inhibits invasion and metastasis of colon cancer cells by enhancing microRNA‐124‐mediated suppression of STAT3" was retracted in 2022. Reasons: duplicated images; signs of a paper mill.

In this study we further found that HIFU induced the mRNA expression of miR‐124 both *in vitro* and *in vivo*. MiRNAs have been shown to play a critical role in regulating metastatic progression, with some miRNAs identified as promoters of metastasis and some identified as suppressors 5. A previous study found that miR‐124 inhibited cell migration in glioma by down‐regulating the expression of Smad2, a critical molecule involved in transforming growth factor β signaling transduction in metastasis regulation 9. The effects of miR‐124 in suppressing cell migration and invasion were also observed in bladder cancer cells and in lung adenocarcinoma cells 15, 16. Consistent with these results, we found that miR‐124 inhibited HCT‐116 cell migration. We also found that miR‐124 inhibitor reversed the effect of HIFU in reducing cell migration. These results indicated that the effect of HIFU in reducing cell migration is via up‐regulating miR‐124.

MiRNAs are non‐coding RNAs that exert biological function via post‐transcriptional regulation, including mRNA degradation and mRNA translation inhibition, through interacting with the 3′‐UTR of mRNA targets 17. Previous studies have shown that miR‐124 could directly bind to a site on the 3′‐UTR of STAT3 and suppress STAT3 expression *in vitro* 18, 19. Consistent with these results, we found that miR‐124 could down‐regulate STAT3 in HCT‐116 cells through a binding site on the 3′‐UTR. A previous study found that miR‐124 suppressed STAT3 in esophageal cancer cells and at the same time suppressed the downstream genes of STAT3, including B‐cell lymphoma‐extra large (Bcl‐xl) and matrix metalloproteinase 9, resulting in induction of cell apoptosis and suppression of cell invasion 20. MiR‐24 was also found to suppress the growth of colorectal cancer by inhibiting STAT3 both *in vitro* and in animal models 19. Taken together, these results suggested an involvement of STAT3 in the function of miR‐124 in cancers.

The article "High‐intensity focused ultrasound inhibits invasion and metastasis of colon cancer cells by enhancing microRNA‐124‐mediated suppression of STAT3" was retracted in 2022. Reasons: duplicated images; signs of a paper mill.

Studies have shown that Janus kinase (JAK)–STAT3 signaling plays a critical role in regulating cell invasion and metastasis 21. STAT3 is a transcription factor whose transcriptional activity is dependent on phosphorylation by JAKs. JAKs phosphorylate STAT3 at Tyr705 residues, facilitating the relocation of STAT3 to the nucleus where dimerized STAT3 binds specific sequences to regulate target genes 22. It was shown that STAT3 could promote tumor metastasis by regulating genes involved in the metastatic process, including down‐regulating E‐cadherin to facilitate the loss of cell to cell contact, up‐regulating Wiskott–Aldrich syndrome protein family member 3 (WASF3) to facilitate actin cytoskeleton reorganization, and regulating a variety of growth factors and cytokines 21. Overactivation of STAT3 is frequently observed in a variety of tumors 23. Previous studies found that the protein levels of both unphosphorylated and phosphorylated STAT3 are significantly increased in invasive colorectal cancer tissues 24. Similarly, constitutive STAT3 activity was also observed in dedifferentiated cancer cells and infiltrating lymphocytes in colorectal cancer samples 25. On the other hand, targeting the aberrant STAT3 activation was considered as a potential treatment for cancer. A previous study showed that suppression of phosphorylated STAT3 by a specific antisense oligonucleotide reduced migration of hepatocellular carcinoma cells, suppressed lung metastasis of orthotopically xenografted hepatocellular carcinoma and prolonged survival time of the model mice 26. As expected, our results showed that HIFU treatment resulted in decreased STAT3 expression and activation, along with suppressed tumor cell metastasis, suggesting that the anti‐metastatic effect of HIFU was via regulating miR‐124–STAT3 signaling. Further studies are warranted to investigate the downstream target of this signaling pathway after HIFU treatment.

It is worth noting that there are several limitations to the current study. First, only one cell line was employed for the observations. It would be more convincing if similar results could be derived in other colon cell lines, even in other types of cancer cells. Second, although various durations of HIFU treatment were applied, its intensity remained the same. Different HIFU intensities could be included in the future study.

The article "High‐intensity focused ultrasound inhibits invasion and metastasis of colon cancer cells by enhancing microRNA‐124‐mediated suppression of STAT3" was retracted in 2022. Reasons: duplicated images; signs of a paper mill.

## Conclusion

We found that HIFU could inhibit metastasis of colon cancer cells in this study. We also confirmed that miR‐124 could directly target STAT3 and the anti‐metastatic effect of HIFU was possibly via up‐regulating miR‐124 and thus suppressing the expression and activation of STAT3.

## Conflict of interest

The authors declare no conflict of interest.

## Author contributions

All authors participated in the design, interpretation of the studies, analysis of the data, and review of the manuscript. MYL and GSW contributed equally to this work. MYL, GSW, HJY, and WX conducted the experiments; HJY and WX wrote the manuscript.
